The article "Metallic Ions Encapsulated in Electrospun Nanofiber for Antibacterial and Angiogenesis Function to Promote Wound Repair" was retracted in 2022. Reasons: original data or images not available; concerns about the data.

# Metallic Ions Encapsulated in Electrospun Nanofiber for Antibacterial and Angiogenesis Function to Promote Wound Repair

**DOI:** 10.3389/fcell.2021.660571

**Published:** 2021-03-25

**Authors:** Chenxi Zhu, Runfeng Cao, Yu Zhang, Ru Chen

**Affiliations:** ^1^Department of Breast Surgery, Hainan General Hospital, Hainan Medical University, Haikou, China; ^2^Department of Dermatology, Xinhua Hospital Affiliated to Shanghai Jiao Tong University School of Medicine, Shanghai, China; ^3^Department of Cardiothoracic Surgery, Shanghai Children’s Hospital, Shanghai Jiao Tong University, Shanghai, China

**Keywords:** electrospinning, silver, magnesium, angiogenesis, antibacterial, wound healing

## Abstract

Electrospun nanofiber is an attractive biomaterial for skin tissue engineering because it mimics the natural fibrous extracellular matrix structure and creates a physical structure suitable for skin tissue regeneration. However, endowing the nanofibrous membranes with antibacterial and angiogenesis functions needs to be explored. In the current study, we aimed to fabricate gelatin/polycaprolactone (GT/PCL) (GT/PCL-Ag-Mg) nanofibers loaded with silver (Ag) and magnesium (Mg) ions for antibacterial activity and pro-angiogenesis function for wound repair. The fabricated GT/PCL membranes had a nanofibrous structure with random arrangement and achieved sustained release of Ag and Mg ions. *In vitro* results indicated that the GT/PCL-Ag-Mg membranes presented satisfactory cytocompatibility with cell survival and proliferation. In addition, the membranes with Ag demonstrated good antibacterial capacity to both gram-positive and gram-negative bacteria, and the Mg released from the membranes promoted the tube formation of vascular endothelial cells. Furthermore, *in vivo* results demonstrated that the GT/PCL-Ag-Mg membrane presented an accelerated wound healing process compared with GT/PCL membranes incorporated with either Ag or Mg ions and pure GT/PCL alone. Superior epidermis formation, vascularization, and collagen deposition were also observed in GT/PCL-Ag-Mg membrane compared with the other membranes. In conclusion, a multifunctional GT/PCL-Ag-Mg membrane was fabricated with anti-infection and pro-angiogenesis functions, serving as a potential metallic ion-based therapeutic platform for applications in wound repair.

## Introduction

As the first barrier to bacterial invasion, skin tissue also modulates body temperature and percepts noxious stimulation (Rahmani Del Bakhshayesh et al., 2018). Skin tissue has a self-healing function after damage by trauma and burns, which is mainly mediated by three overlapping processes: inflammation, proliferation, and remolding (Xie et al., 2021). However, some specific circumstances, such as large area skin defects or skin trauma in aging patients, cannot self-heal sufficiently to achieve structural and functional repair of the damaged skin tissue (Qu et al., 2019). Delayed or incomplete skin repair will increase the risk of bacterial infection, increasing the psychological and physical burden of patients (Wang Z. J. et al., 2021). Therefore, developing wound care products that improve healing and prevent complications is needed in clinical practice.

Wound dressings, an important factor for skin tissue engineering, have been widely explored and applied to wound healing (Xuan et al., 2020). Ideal wound dressings should mimic the native extracellular matrix (ECM) structure to provide cell adhesion, proliferation, and migration, promoting the skin tissue healing process (Chen et al., 2017). Electrospinning technologies have been widely used to produce nanofibers to mimic the topographical structure of collagen fibers in skin tissue given its cost effectiveness and versatility (Liu et al., 2017; Miguel et al., 2018). The fabricated nanofibers have advantages of a high surface-to-volume ratio, excellent mechanical property, and high porosity (Lin et al., 2020). However, the ECM-like nanofibrous structure is limited to the cell–biomaterial interaction and how to further modulate the wound healing process remains to be studied (Choi et al., 2008; Lai et al., 2014). Angiogenesis plays an important role during wound healing. Modulation of angiogenesis would boost the wound healing processing, reducing the healing time (Zhu et al., 2019). In addition to the faster wound closure, preventing wound infections, which often occurs during wound healing, negatively impacting the healing process, is also important (Albright et al., 2018). Several growth factors, drugs, or nanoparticles, such as Ag nanoparticles and vascular endothelial cell growth factor (VEGF), have been incorporated into electrospun fibers to build a controlled-release system to modulate these two processes (Xie et al., 2013; Tra Thanh et al., 2018).

Metal cations, which are involved in a wide range of biological processes, play an important role in the human body (Mushahary et al., 2013; Bi et al., 2019). Silver (Ag) iron has being studied as an antibacterial agent because of its broad-spectrum antibacterial properties (Nhi et al., 2016). Furthermore, Ag can avoid the bacterial resistance caused by the use of traditional antibiotics. However, growth factors or drugs are often used for angiogenesis, which is accompanied by organic component deactivation (Vijayan et al., 2019). As a result, establishing an inorganic ion therapy platform with angiogenesis and anti-infection still needs to be explored. Magnesium (Mg) and its alloys have been applied to orthopedic implants because of their osteogenesis and angiogenesis function (Han et al., 2020). A previous study showed that Mg can significantly promote angiogenesis-related gene expression, including HIF-1α and VEGF, and enhance the blood vessel formation (Gao et al., 2020). However, whether Mg can be incorporated into electrospun nanofibers to promote vascularization remains unknown. In the present study, both Ag and Mg were incorporated into electrospun nanofibers to simultaneously endow the nanofibers with anti-infection and pro-angiogenesis properties.

Therefore, the objective of the current study was to develop an inorganic metallic ion therapy platform based on electrospun nanofibers to prevent bacterial infection and promote angiogenesis, enhancing the wound healing process and reducing the healing time. Ag was incorporated to achieve the anti-infection function of fibers, while Mg was incorporated to achieve a pro-angiogenesis function. The *in vitro* biocompatibility, pro-angiogenesis, and anti-infection functions of Ag and Mg-incorporated gelatin/polycaprolactone (GT/PCL-Ag-Mg) membranes were evaluated. Furthermore, the therapy efficiency of the GT/PCL-Ag-Mg membrane to promote healing of the bacterial infected wounds were performed. The whole experimental design is illustrated in Scheme 1.

**SCHEME 1:** The overall experimental design. A GT/PCL nanofiber membrane with Ag and Mg ions (GT/PCL-Ag-Mg) was fabricated, and its antibacterial and angiogenesis function were verified using *in vitro* and *in vivo* studies.

## Materials and Methods

### Fabrication of the GT/PCL-Based Nanofibrous Membranes

Four electrospun solutions were prepared for printing different membranes: pure GT/PCL, GT/PCL-Ag, GT/PCL-Mg, and GT/PCL-Ag-Mg.

GT/PCL solution: GT (Sigma) and PCL (Sigma) were dissolved in a mass ratio of 50/50 in hexafluoroisopropanol (Aladdin) at a concentration of 10% w/v.

GT/PCL-Ag solution: 10.2 mg of AgNO_3_ was uniformly dispersed in 10 mL of the GT/PCL solution.

GT/PCL-Mg solution: 10.2 mg of MgCl_2_ was uniformly dispersed in 10 mL of the GT/PCL solution.

GT/PCL-Ag-Mg solution: 10.2 of mg AgNO_3_ and 10.2 mg of MgCl_2_ were uniformly dispersed in 10 mL of the GT/PCL solution.

Nanofibrous membrane fabrication: the four electrospun solutions were delivered at a feeding rate of 1.5 mL/h by a syringe pump (KDS100, KD Scientific) to a blunt medical metal needle (22G) used as the spinneret. A potential of 13.0 kV from a high-voltage power supply (TXR1020N30-30, Teslaman, Dalian, China) was applied between the spinneret and a grounded aluminum foil (200 mm × 200 mm) mounted on the surface of an adjustable lab jack, stationed 12 cm from the tip of the spinneret. The prepared nanofibrous membranes were dried in a vacuum oven overnight at room temperature to remove residual solvent and cross-linked in an airtight container with 25% glutaraldehyde vapor for 30 min (Yan et al., 2021). The prepared membranes were sterilized for 30 min under UV irradiation and then trimmed into different shapes for subsequent use.

### Morphological Observation

The macro-morphologies of the prepared membranes were photographed using a digital camera and a digital vacuum scanning electron microscope (SEM, JEOL JSM-5600LV, Japan). Samples were critical-point dried and then examined using the SEM (Xu et al., 2020).

### Elemental Mapping Analysis

The elemental mapping results of the electrospun membranes were obtained using an energy dispersive spectrometer (EDS, OXFORD MAX-80, INCA SYSTEM).

### FTIR Spectroscopic Analysis

The formation of Ag, Mg, GT/PCL, GT/PCL-Ag, GT/PCL-Mg, and GT/PCL-Ag-Mg were analyzed with Fourier transform infrared (FTIR) spectroscopy using ATR–FTIR (model-Alpha, Bruker, Germany) spectrometer, scanning from 250 to 4,000 cm^–1^ at room temperature.

### *In vitro* Release of Ag and Mg

Membranes with a diameter of 10 mm were immersed in 500 mL deionized water at 37°C for 1, 4, 7, 10, 13, 16, 19, and 22 days to measure the release of Ag and Mg ions from GT/PCL-Ag-Mg. The deionized water was refreshed at each time point. The concentrations of Ag and Mg in the collected deionized water were determined using inductively coupled plasma atomic emission spectrometry (ICP-AES, PerkinElmer Optima 7000 DV).

### Cytocompatibility

To evaluate the cytocompatibility of the nanofibrous membranes, five experimental groups, GT/PCL, GT/PCL-Ag, GT/PCL-Mg, and GT/PCL-Ag-Mg, as well as a Control group without membranes were evaluated. Fibroblasts obtained from the Type Culture Collection of the Chinese Academy of Sciences were incubated at 37°C in a 5% CO_2_ atmosphere. After culture and expansion for two passages, the fibroblast suspension at a density of 2 × 10^5^ cells mL^–1^ was seeded onto the membranes. A culture dish was used as the Control group. After 1 and 4 days of culture, the fibroblast viability on each membrane was evaluated using the Live and Dead Cell Viability Assay (Invitrogen, United States) following the manufacturer’s instructions, and the samples were examined using a confocal microscope (Nikon, Japan). The fibroblast viability was also measured using a cell counting kit-8 (CCK-8; Dojindo, Japan) following the manufacturer’s instructions, and the optical density (OD) was measured at 450 nm (Xu et al., 2020).

### Antibacterial Performance

*Escherichia coli* (*E. coli*) and *Staphylococcus aureus* (S. *aureus*) were used for the antibacterial evaluations. These bacteria were incubated in Luria Bertani (LB) liquid medium under constant stirring. After the OD600 value reached 2.0, 10 mL of the bacterial fluid was centrifuged at 3,000 rpm for 10 min to remove the medium. The obtained bacteria precipitate was resuspended in 10 mL PBS. Nanofibrous membranes were cut into 2 cm × 2 cm pieces and then incubated with 1 mL of the bacterial suspension for 5 h. The obtained bacterial solution was diluted with PBS to a concentration range of 10^–4^ to 10^–6^, and 100 μL of the solution was homogeneously seeded in dishes with LB medium. After incubation at 37°C overnight, images of the LB dishes were captured, and the number of bacterial colonies was counted. Three independent samples were analyzed. The inhibition rate (%) was calculated using: (α − β)/α × 100%, where α and β refer to the average colony number in the blank control and samples, respectively.

### Tubular Formation Assay

An *in vitro* tubular formation assay was performed using Matrigel (BD Bioscience) according to the manufacturer’s specifications. Human umbilical vein endothelial cells (HUVECs) were purchased from the Type Culture Collection of the Chinese Academy of Sciences and seeded into 24-well plates coated with Matrigel, and different membranes were added. After 6 h, the cells were imaged (Chen et al., 2019).

### *In vivo* Wound Healing

To access the antibacterial wound healing property of the samples, we built an infectious full-thickness wound model on the backs of male Sprague Dawley rats (6–8 weeks, weight: 180–220 g). The mice were purchased from Shanghai SLAC Laboratory Animal Co., Ltd. (Shanghai, China). All animal procedures were approved by the Institutional Animal Care and Use Committee of Shanghai Jiao Tong University School of Medicine. The mice were randomly divided into five groups (*n* = 3 per group). The excised circle wounds (10 mm in diameter) were covered without nanofibrous membranes (served as a control group) or with GT/PCL, GT/PCL-Ag, GT/PCL-Mg, and GT/PCL-Ag-Mg nanofibrous membranes fixed with an elastic adhesive bandage and left untreated. The wounds were photographed at 1, 7, and 14 days post-operation. The wound healing rate was calculated by the following equation: (W_0_-W_*t*_)/W_0_ × 100%, where W_0_ is the wound size at Day 0 and W_*t*_ is time interval “t.”

### Histopathological Analyses

Tissue samples from the wounds were harvested and fixed with 4% paraformaldehyde, dehydrated, embedded in paraffin, and cut into 5-μm thick slices. The slices were stained with hematoxylin and eosin (HE). Masson’s trichrome and Sirius red staining were used to further evaluate the fibrotic remodeling. The *in vivo* bacteria were evaluated by FISH staining (Atieh et al., 2013). Angiogenesis was evaluated by immunohistochemical staining of CD31, as previously described (Shi et al., 2017). The HE, Masson’s trichrome, FISH, and CD31 staining images were analyzed with ImageJ software to quantitatively analyze the extent of epidermis thickness, collagen fiber percentage, amount of bacteria, and vascularization.

### Statistical Analysis

All quantitative data are shown as mean ± standard deviation from at least three specimens. One-way analysis of variance was used to evaluate the statistically significant differences between groups. Data were analyzed using SPSS17.0. *p* < 0.05 was considered statistically significant.

## Results and Discussion

### Characterization of the Fabricated Membranes

Electrospun technology has been widely applied in skin tissue engineering because of several fundamental features beneficial for rapid and functional wound healing and regeneration (Aavani et al., 2019). The biomimetic ECM nanofibrous architecture provides a platform for suitable cell–material interactions and material structure based intracellular signaling pathway activation (Iacob et al., 2020). In addition, the nanopores within the electrospun membranes can increase the nutrient and waste exchange, and form a physical barrier to resist bacterial infection. In the present study, gelatin and PCL were used to fabricate the nanofibers because of their good cytocompatibility, superior mechanical property, and adjustable biodegradability (Yan et al., 2021). Our results revealed that the GT/PCL nanofibers were successfully fabricated with random arrangement using well-established electrospinning conditions (Figure 1). In addition, Ag was added to endow antibacterial property, while Mg was added to endow the pro-angiogenesis property of the GT/PCL-AG-Mg membrane. As shown in Figures 1A,B, the incorporation of Ag or Mg ions did not affect the morphology and nanofibrous structure of the membranes. Elemental mapping (Figure 1C) and FTIR (Figure 1D) analyses further confirmed the successful encapsulation of Ag and Mg ions in the GT/PCL-Ag-Mg membranes. The releasing rate of Ag and Mg was further evaluated. As shown in Figures 1E,F, the Ag and Mg ions were gradually released from the GT/PCL-Ag-Mg membranes over time.

**FIGURE 1:** Characterizations of the nanofibrous membranes. **(A)** Gross and **(B)** SEM images of the fabricated GT/PCL, GT/PCL-Ag, GT/PCL-Mg, and GT/PCL-Ag-Mg membranes. **(C)** Mapping of carbon, Ag, and Mg elements in GT/PCL-Ag-Mg membrane. **(D)** FTIR analysis for Ag and Mg ions, as well as GT/PCL, GT/PCL-Ag, GT/PCL-Mg, and GT/PCL-Ag-Mg membranes. The releasing rate of **(E)** Ag and **(F)** Mg in the GT/PCL-Ag-Mg membrane.

### Cytocompatibility Evaluation of the Fabricated Membranes

The cytocompatibility of the fabricated membranes were evaluated by live and dead staining and CCK-8 tests of fibroblasts. The live and dead staining results showed that fibroblasts were viable on all control, GT/PCL, GT/PCL-Ag, GT/PCL-Mg, and GT/PCL-Ag-Mg groups (Figure 2A). Cells spread out with polygonal morphology on all membranes at 4 days. The CCK-8 test was performed to assess the cell proliferation on the membranes and evaluate the effect of released ions on the proliferation rate of the cells. As shown in Figure 2B, no obvious difference was observed between the fibroblasts seeded in the Control, GT/PCL, GT/PCL-Ag, GT/PCL-Mg, or GT/PCL-Ag-Mg groups. Ag nanoparticles can accumulate within human keratinocytes and mouse fibroblasts, causing DNA damage and cell apoptosis (Jiravova et al., 2016). In the current study, we used Ag ion-releasing nanofibrous membranes to endow the scaffolds with excellent antibacterial function. Results showed that the Ag released from membranes caused no toxic effect on the variability and proliferation of fibroblasts. Furthermore, a previous study showed that Ag ions can replace Ag nanoparticles to achieve antimicrobial properties and maintain cell variability and proliferation (Mohiti-Asli et al., 2014). For Mg ions, the study showed that Mg primarily affected the adhesion and migration behavior of human gingival fibroblasts instead of proliferation (Amberg et al., 2018; Wang L. Y. et al., 2021). In the present study, no impaired variability or increased proliferation rate of the fibroblasts were observed.

**FIGURE 2:** Cytocompatibility of nanofibrous membranes. **(A)** Live and dead staining of fibroblasts cultured *in vitro* and **(B)** proliferation indicated by CCK-8 on Control, GT/PCL, GT/PCL-Ag, GT/PCL-Mg, and GT/PCL-Ag-Mg groups at 1 and 4 days. NS, no statistical difference.

### Antibacterial and Pro-angiogenesis Properties of the Fabricated Membranes

#### Antibacterial Function

Antibacterial behavior is critical for skin tissue engineering and also conducive to accelerating the wound healing process (Qu et al., 2018). The antibacterial property of GT/PCL membranes with different kinds of ions were evaluated against *E. coli* and *S. aureus in vitro*. *E. coli* is a gram-negative bacterium with rod shape, while *S. aureus* is a gram-positive bacterium with a coccal shape (Yasuyuki et al., 2010). The inappropriate use of antibiotics and disinfectants has led to the emergence of antibiotic-resistant bacteria, even multi-drug resistant bacteria (Hemlata et al., 2017). Therefore, reducing the use of antibiotics and finding an effective alternative are important for clinical practice. Ag is an attractive alternative to antibiotics because of its excellent property against a wide range of pathogens (Zheng et al., 2019) and has been widely used in medical products, such as wounds dressing and catheters, to inhibit the bacteria growth (Rtimi et al., 2016; Dissemond et al., 2020). As shown in Figures 3A,B, GT/PCL groups with Ag (including GT/PCL-Ag and GT/PCL-Ag-Mg membranes) significantly inhibited the growth of *E. coli* and *S. aureus*. In contrast, the incorporation of Mg (including GT/PCL-Mg and GT/PCL-Ag-Mg groups) had no anti-bacterial effect for either *E. coli* or *S. aureus*. Moreover, statistical analyses showed that GT/PCL membranes containing Ag significantly inhibited the survival rate of *E. coli* (Figure 3D) and *S. aureus* (Figure 3E). The incorporation of Ag endowed antibacterial function to the electrospun GT/PCL membranes (Xing et al., 2010). Although complete understanding of the underlying antibacterial mechanism of Ag ions is not clear, several studies have indicated that the antibacterial function may be attributed to the following factors: (1) released Ag ions with a positive charge can interact with the negatively charged cell membrane, causing structural changes and interfering with its integrity; (2) the intracellular Ag ions can interact with the thiol (sulfhydryl) groups in enzymes and proteins (Feng et al., 2000; Kedziora et al., 2018). For example, Ag can affect the respiration chain, leading to consumption of intracellular NADPH and reactive oxygen species (ROS) accumulation. The increased ROS level will induce elevated intracellular oxidative stress and cause oxidative damage to the cell structure such as DNA and lipids (Jung et al., 2008).

**FIGURE 3:** *In vitro* antibacterial and pro-angiogenesis properties evaluations. Amount of **(A)** *E. coli* and **(B)** *S. aureus* on agar plates after incubation for 24 h on Control, GT/PCL, GT/PCL-Ag, GT/PCL-Mg, and GT/PCL-Ag-Mg groups. **(C)** Tube formation of HUVECs *in vitro* on Control, GT/PCL, GT/PCL-Ag, GT/PCL-Mg, and GT/PCL-Ag-Mg groups. Survival rate of **(D)** *E. coli* and **(E)** *S. aureus* on each group. Statistical analyses of tube **(F)** formation numbers and **(G)** branch points for each group. ^∗^*p* < 0.05.

#### Pro-angiogenesis Function

Skin tissue is highly vascularized; therefore, early rebuilding of the vascularization is essential for skin tissue regeneration. The lack of blood supply and nourishment will delay the wound healing process, and also increase the infection risk (Bi et al., 2019). Mg is widely applied in bone tissue engineering, as it can increase the osteogenesis and pro-angiogenesis properties of bone scaffolds (Zheng et al., 2020), and increase the proliferation of endothelial cells (Shigematsu et al., 2018). A previous study showed that a Mg-coated Ti6Al4V scaffold promoted angiogenesis by increasing the gene expression and secretion of angiogenic factors such as the HIF-1α and VEGF (Gao et al., 2020). Furthermore, Mg can enhance the synthesis of nitric oxide, which is involved in the angiogenesis process. A tube formation test was performed to observe the effect of GT/PCL membranes with different incorporated ions on the *in vitro* tubulogenesis ability of HUVECs. It has been shown that magnesium with concentration between 1 and 5 mM, especially 5 mM, promoted the angiogenic ability of HUVECs (Liu et al., 2020). Low concentrations of Mg ions (<10 mM) increased cell viability, proliferation rate, cell spreading and migration rate, while high concentrations of Mg ions (40–60 mM) have deleterious effect (Ma et al., 2016). Therefore, in present study, the concentration of Mg in electrospun nanofibers was approximately 10 mM. With the degradation of electrospun nanofibers, the Mg ions was gradually released, which is lower than 10 mM. Consistent with previous studies, our results showed that GT/PCL-Mg and GT/PCL-Ag-Mg significantly promoted the tube formation (Figures 3C,F) and vessel branch points (Figure 3G), indicating that GT/PCL membranes with Mg exhibited the potential of angiogenesis.

### *In vivo* Animal Study

After the *in vitro* antibacterial and pro-angiogenesis function were verified, the fabricated GT/PCL nanofibrous membranes were used to treat round, full-thickness skin defects infected with bacteria to investigate the wound healing performance of the scaffolds. Figure 4A demonstrates that the gross images of the wound closure condition 1, 7, and 14 days after treatment with GT/PCL, GT/PCL-Mg, GT/PCL-Ag, and GT/PCL-Ag-Mg and without any membranes (Control group). The wound area of all groups decreased with increasing time; however, wounds treated with GT/PCL loaded with Ag, Mg, or both exhibited fast healing at the same time point (Figure 4A). In terms of the wound healing rate, GT/PCL loaded with Ag or Mg showed significant higher healing than pure GT/PCL membranes or the Control group at 7 and 14 days (Figure 4C). The GT/PCL-Ag-Mg group showed a 71.3 ± 2.9% wound healing rate at 7 days, whereas the Control and GT/PCL group only obtained 34.3 ± 1.7 and 35.7 ± 2.8%, respectively (Figure 4C). At 14 days, nearly the whole wound area was filled with neo-tissue in GT/PCL-Ag-Mg with only a smaller scar remaining, indicating better wound healing outcomes than the other groups (Figure 4C). Our results showed that the incorporation of Ag or Mg significantly promoted the healing process of wounds compared with Control or pure GT/PCL membranes. In addition, the GT/PCL-Ag-Mg membrane achieved optimal therapeutic effect.

**FIGURE 4:** Gross and HE staining evaluations of wound healing. **(A)** Gross observations of wound healing at 1, 7, and 14 days on the Control, GT/PCL, GT/PCL-Ag, GT/PCL-Mg, and GT/PCL-Ag-Mg groups. **(B)** HE staining of repaired tissue at 7 and 14 days on the Control, GT/PCL, GT/PCL-Ag, GT/PCL-Mg, and GT/PCL-Ag-Mg groups. Quantitative analyses of **(C)** wound healing rate at 7 and 14 days and **(D)** epidermis thickness of repaired tissue on Control, GT/PCL, GT/PCL-Ag, GT/PCL-Mg, and GT/PCL-Ag-Mg groups. ^∗^*p* < 0.05.

Histological analysis was further adopted to evaluate the regeneration quality of the repaired skin tissue. HE staining showed that epidermal structure was formed for GT/PCL membranes loaded with either Ag or Mg ions or both at the early timepoint of 7 days (Figure 4B). At 14 days, partial epidermis formed in the Control group and pure GT/PCL membranes. Alternatively, for the GT/PCL-Ag-Mg group, the epidermis length and thickness obviously increased from 7 days and was greater than the other groups (Figures 4B,D). Normal epidermal and dermal junctions were also observed in the GT/PCL-Ag-Mg groups, including epidermal protrusions and dermal projections.

Masson’s trichrome staining and Sirius red staining were further performed to observe the collagen deposition in the wounds treated with different nanofibrous membranes (Figure 5). Collagen fiber was stained blue with Masson’s trichrome staining. As shown in Figure 5A, intensive blue stained collagen fibers were observed in the GT/PCL-Ag-Mg groups while less collagen deposition was in the GT/PCL-Mg groups at 7 days. However, nearly no collagen fibers were observed at 7 days in the other groups. At 14 days, the deposition of collagen was observed in all groups. However, the dermal collagen in the Control, GT/PCL, and GT/PCL-Ag groups was disorganized and sparse. Alternatively, the collagen in GT/PCL-Mg and GT/PCL-Ag-Mg was bundled and arranged in a regular pattern (Figure 5A). As shown in Figure 5B, Sirius red staining also confirmed abundant collagen fiber formation and deposition in the ECM. Sirius red staining can reflect the major deposited collagen fiber type, as collagen type III stains green and type I stains red (Bo et al., 2020). In natural dermal tissue, the predominant collagen is type I. Therefore, the abundant deposition of collagen I in repaired skin tissue represents successful wound healing. At 7 days, the collagen type was primarily type III in all groups, with the exception of more type I in wounds treated with the GT/PCL-Ag-Mg membranes (Figure 5B). With the remodeling of regenerated skin tissue, collagen type I fiber increases and replaces collagen type III. In hypertrophic scars, the predominant collagen type is III (Cuttle et al., 2005; Li et al., 2015). Our results showed that collagen type I increased with time in all groups. However, for GT/PCL loaded with metallic ions, an increase in collagen type I/III was observed. The satisfactory collagen deposition is related with the pro-angiogenesis and anti-infection function of Ag or Mg ions in the GT/PCL membranes.

**FIGURE 5:** Evaluation of the collagen regeneration. **(A)** Masson’s trichrome and **(B)** Sirius red staining of repaired skin tissue at 7 and 14 days on Control, GT/PCL, GT/PCL-Ag, GT/PCL-Mg, and GT/PCL-Ag-Mg groups. Collagen fiber percentage of repaired tissue at 7 and 14 days on Control, GT/PCL, GT/PCL-Ag, GT/PCL-Mg, and GT/PCL-Ag-Mg groups **(C)**. Scale bar: 100 μm. ^∗^*p* < 0.05.

FISH staining was performed to detect the pathogen in the wound area (Figure 6A). The results show that a large number of pathogens were observed in the Control and GT/PCL groups. The incorporation of Ag within GT/PCL membranes significantly inhibited the growth of pathogens, while the GT/PCL-Mg showed limited anti-infection ability at 3 days (Figure 6C). Furthermore, angiogenesis is an important process in the healing of a wound and the functional restoration of skin tissue. Impaired vascularization will delay the closure of a wound area and increase the infection risk. CD31 immunohistochemical staining was further adopted to evaluate the vascularization of regenerated neo-tissue (Figure 6B). At 7 days, obvious CD31 positive vessels were observed in the Mg-loaded GT/PCL membranes. With an increase of healing time, the vascularization increased in all groups, especially for GT/PCL membranes with Mg ions. The average number of vessels per field in the GT/PCL-Mg and GT/PCL-Ag-Mg membranes is nearly triple that of the Control group (Figure 6D). In conclusion, our results showed that Ag and Mg ions loaded into GT/PCL membranes can achieve satisfactory wound healing outcomes with abundant collagen deposition (mainly collagen type I), simultaneous antibacterial function, with an abundant neovascularization formation.

**FIGURE 6:** *In vivo* antibacterial and pro-angiogenesis properties evaluations. **(A)** FISH staining of bacteria at 3 days on Control, GT/PCL, GT/PCL-Ag, GT/PCL-Mg, and GT/PCL-Ag-Mg groups. **(B)** CD31 staining of repaired skin tissue at 7 and 14 days on Control, GT/PCL, GT/PCL-Ag, GT/PCL-Mg, and GT/PCL-Ag-Mg groups. Quantitative analyses of **(C)** bacterial counts and **(D)** neovascularization in repaired tissue at 7 and 14 days on Control, GT/PCL, GT/PCL-Ag, GT/PCL-Mg, and GT/PCL-Ag-Mg groups. ^∗^*p* < 0.05.

## Conclusion

In this study, we prepared a GT/PCL membrane with ECM-biomimetic structure using electrospinning technology, incorporating Ag and Mg ions into the membrane to establish a metallic ion based therapy platform to achieve simultaneous antibacterial function and pro-angiogenesis. *In vitro* antibacterial and angiogenesis studies showed that Ag and Mg ions loaded into the GT/PCL membranes significantly inhibited the growth of *E. coli* and *S. aureus* pathogens, and promoted the tube formation of HUVECs. Furthermore, *in vivo* results showed that GT/PCL-Ag-Mg membranes obtained superior wound repair outcomes compared with other groups, as indicated by the wound closure area, epidermis formation, collagen deposition, and vascularization. In conclusion, we established a multifunction platform with anti-infection and pro-angiogenesis properties by incorporating Ag and Mg metallic ions into GT/PCL nanofibrous membranes for potential application to clinical skin defects.

## Data Availability Statement

The raw data supporting the conclusions of this article will be made available by the authors, without undue reservation.

## Ethics Statement

All animal procedures were approved by the Institutional Animal Care and Use Committee of Shanghai Jiao Tong University School of Medicine.

## Author Contributions

CZ: scaffolds design, culture cells, and animal operation. RCa: data analyses and manuscript revises. YZ: data analyses. RCh: funding acquisition and review and editing. All authors contributed to the article and approved the submitted version.

## Conflict of Interest

The authors declare that the research was conducted in the absence of any commercial or financial relationships that could be construed as a potential conflict of interest.
